The article "Superparamagnetic Nanoparticles for Atherosclerosis Imaging" was published in 2014. Journal: Nanomaterials (Basel).

# Superparamagnetic Nanoparticles for Atherosclerosis Imaging

**DOI:** 10.3390/nano4020408

**Published:** 2014-06-05

**Authors:** Fernando Herranz, Beatriz Salinas, Hugo Groult, Juan Pellico, Ana V. Lechuga-Vieco, Riju Bhavesh, J. Ruiz-Cabello

**Affiliations:** 1 Advanced Imaging Unit, Department of Epidemiology, Atherothrombosis and Imaging, Spanish National Centre for Cardiovascular Research (CNIC), Melchor Fernández Almagro, 3, 28029 Madrid, Spain; E-Mails: beachinchilla@gmail.com (B.S.); hugo.groult@externo.cnic.es (H.G.); jpellico@externo.cnic.es (J.P.); anavictoria.lechuga@cnic.es (A.V.L.-V.); riju.bhavesh@cnic.es (R.B.); ruizcabe@cnic.es (J.R.-C.); 2 CIBER of Pulmonary Diseases, Biomedical Research Network, Carlos III Health Institute, 28029 Madrid, Spain; 3 Department of Physicochemistry II, Faculty of Pharmacy, Complutense University Madrid (UCM), Plaza Ramón y Cajal s/n Ciudad Universitaria, 28040 Madrid, Spain

**Keywords:** iron oxide nanoparticles, cardiovascular imaging, atherosclerosis plaque, chemoselective functionalization

## Abstract

The production of magnetic nanoparticles of utmost quality for biomedical imaging requires several steps, from the synthesis of highly crystalline magnetic cores to the attachment of the different molecules on the surface. This last step probably plays the key role in the production of clinically useful nanomaterials. The attachment of the different biomolecules should be performed in a defined and controlled fashion, avoiding the random adsorption of the components that could lead to undesirable byproducts and ill-characterized surface composition. In this work, we review the process of creating new magnetic nanomaterials for imaging, particularly for the detection of atherosclerotic plaque, *in vivo*. Our focus will be in the different biofunctionalization techniques that we and several other groups have recently developed. Magnetic nanomaterial functionalization should be performed by chemoselective techniques. This approach will facilitate the application of these nanomaterials in the clinic, not as an exception, but as any other pharmacological compound.

## 1. Introduction

Superparamagnetic iron oxide nanoparticles (IONPs) are entering a new phase in the biomedical field, with a mushrooming spectrum of applications that no longer limits its clinical use [1]. For instance, oncological research has widely found an application of these nano-platform-based diagnosis and therapy tools, due to their specific features [2,3]. The situation for cardiovascular diseases is not that advanced yet; but, the research is quite intensive, and most researchers working in the field have realized the potential of applying nanotechnology to their work. This has translated into many results in conditions, like atherosclerotic plaque, stroke or myocardial infarction [4,5,6,7,8].

The article "Superparamagnetic Nanoparticles for Atherosclerosis Imaging" was published in 2014. Journal: Nanomaterials (Basel).

**Figure 1:** Steps in the synthesis of iron oxide nanoparticles (IONP) for preclinical atherosclerosis imaging. (**A**) Mixture of iron precursors and different surfactants in organic solvents; (**B**) Iron oxide nanoparticles in organic solvent; (**C**) Phase transfer to a water-based solution, in two steps or in a one-step phase transfer and functionalization (red arrow); (**D**) Functionalization of the nanoparticles for selective and/or multifunctional imaging; (**E**) Imaging of atherosclerotic plaque with iron oxide nanoparticles. EPR, enhanced permeability and retention.

The interest in the application of these compounds in cardiovascular imaging and chemical probes, in general, is reflected in the number of reviews dealing with several aspects of the field. Our approach in this review is somehow different, and it is depicted in Figure 1. We will study the different steps allowing for the *in vivo* detection of atherosclerotic plaque. The first step is the combination of iron precursors and surfactants, which includes the selection of the most appropriate combination of compounds and solvent to get nanoparticles with good crystallinity, magnetic and colloidal properties. Next in this process is to get water-stable and functionalized nanoparticles. This has been traditionally done in two steps, a phase transfer reaction and a second step with the attachment of the biomolecule. However, with the development of new approaches that perform chemical reactions over the initial organic surfactant, this process can be reduced to a single step in which the stabilization in water and the attachment of a biologically relevant molecule is done altogether. The final step is the preclinical application of the nanoparticles to an animal model of atherosclerosis. To get the selective accumulation of the nanoparticles inside the body, several strategies can be followed, e.g., macrophage targeting, plaque calcification, the angiogenesis process or by taking advantage of the enhanced permeability and retention (EPR) effect [9].

By studying the different chemical routes for the synthesis of homogeneous superparamagnetic and biofunctionalized IONPs and the biology behind atherosclerosis disease, a rational and focused strategy can be developed for the synthesis of clinically-relevant nanoparticles.

## 2. Synthesis of Iron Oxide Superparamagnetic Nanoparticles

Due to the relevance and wide spectrum of applications with IONPs, there has been a tremendous increase in the synthetic methodologies in the past few years. The most relevant approaches include methods, such as coprecipitation [10,11,12], thermal decomposition [13,14,15], sonolysis [16,17], sol-gel processes [18,19], spray and laser pyrolysis [20,21,22], hydrothermal and high temperature synthesis [23,24,25,26], nanoreactors, such as protein cages [27,28,29], vesicles [30], microemulsions [31,32] and microwave-assisted synthesis [33,34,35,36,37,38]. For the sake of simplicity, we will focus here only on the most interesting ones from the biomedical point of view, particularly the most common ones with a higher prevalence and projection: coprecipitation, thermal decomposition and microwave-assisted synthesis.

The article "Superparamagnetic Nanoparticles for Atherosclerosis Imaging" was published in 2014. Journal: Nanomaterials (Basel).

### 2.1. Co-Precipitation Method

One of the most employed methodologies for the synthesis of iron oxide nanoparticles for biomedical applications is the co-precipitation method. This process involves a reaction of the aqueous mixture of Fe^2+^/Fe^3+^ salt solutions with a base. Under these conditions, magnetite nanoparticles are formed by the aggregation of primary particles within a Fe(OH)_2_ gel. This methodology, developed by Massart *et al.*, was carried out initially without the incorporation of any stabilizing molecule on the surface of the nanoparticles.[10] In this work, they reported the controlled preparation of IONPs through alkaline precipitation of FeCl_3_ and FeCl_2_. The magnetite (Fe_3_O_4_) particles formed were roughly spherical, with a diameter of 8 nm, measured by XRD.

In this approach, magnetite is prepared by adding a base to an aqueous mixture of Fe^2+^ and Fe^3+^ salts in a 1:2 molar ratio. The overall reaction may be written as follows, leading to the precipitation of black magnetite [10]:

Fe^2+^ + 2Fe^3+^ + 8OH^−^ → Fe_3_O_4_ + 4H_2_O

In this reaction, a complete precipitation of Fe_3_O_4_ should be expected at pH 9, while maintaining a molar ratio of Fe^3+^:Fe^2+^ of 2:1. The reaction is performed under a non-oxidizing oxygen-free environment, by bubbling N_2_ in the reaction, something that also helps to reduce the final size of the nanoparticles [39].

A wide variety of parameters must be considered in this method in order to control size, magnetic characteristics and colloidal stability in the solution. Magnetization can vary drastically with synthesis variations even within particles of a similar size, due to the incorporation of impurities into the crystal structure and the involvement of surface effects [40,41]. Generally, magnetization saturation values of magnetite nanoparticles obtained by this method are in the range of 30–50 emu/g; lower than the 90 emu/g reported for their bulk form [42,43]. In addition, the determining parameter in controlling their size is the pH, which must be adjusted in both the synthesis and purification steps. As a result, the production of narrowly dispersed particles remains a significant challenge in this method [44]. Other factors, like adjustment of the Fe^3+^:Fe^2+^ ratios, heating regimes and the coating-iron ratios must be strictly controlled [45,46].

The article "Superparamagnetic Nanoparticles for Atherosclerosis Imaging" was published in 2014. Journal: Nanomaterials (Basel).

After the initial development by Massart *et al.*, the number of coatings that have been used vary from polymers [47,48,49,50], to dendrimers [51] and organic acids [52,53,54]. For example, adding increasing amounts of citrate ions in the Massart process allows for a decrease in the diameter of citrate-coated nanoparticles from 8 to 3 nm. Citrate chelates iron ions, preventing nucleation, and at the same time, the adsorption of citrate on the nuclei produces hydrolysis, inhibiting the growth of the nuclei [55].

The main advantage of the co-precipitation process is that a large amount of water-stable nanoparticles are obtained. However, the control of particle size distribution is limited, because only kinetic factors are controlling the growth of the crystal. This leads to the synthesis of somehow heterogeneous samples in terms of size and shape. Another problem that can be found with this approach is the weak attachment of the surfactant to the surface and the reduced number of functional groups that can be found on the surface, all of this complicating the final functionalization for biomedical applications.

### 2.2. Thermal Decomposition of Organic Precursors

High temperature decomposition of iron organic precursor mixed with surfactants in organic solvents is progressively becoming the standard way for the preparation of IONPs. This method yields nanoparticles of a narrow size distribution, good crystallinity and high magnetization saturation values (Figure 2) [56]. The first synthesis introduced by Aliviastos *et al.* reported the injection of FeCup_3_ (Cup:*N*-nitrosophenylhydroxylamine) solutions in hot trioctylamine resulting in nanoparticles of 4 to 10 nm average diameters as a function of the temperature (250 °C to 300 °C) and the quantity of iron precursor added. A second method consisted of the preparation of iron nanoparticles by the injection of the organic Fe(CO)_5_ precursor in the surfactant mixture followed by an *in situ* oxidation phase to produce highly crystalline and monodispersed maghemite nanoparticles with sizes from 4 to 16 nm [57,58,59]. Although the hot injection technique guarantees instant nucleation and homogenous growth for an optimal quality of the nanoparticles, it also presents drawbacks mainly related to safety and toxicological issues [60]. Heating up processes were then proposed with iron oleate, an intermediate prepared from FeCl_3_ and the mechanisms of crystallizations studied [61,62]. In 2002, Sun *et al.* described a single step synthesis using iron acetylacetonate thermal degradation by progressive heating in diphenyl ether in the presence of alcohol, oleylamine and oleic acid surfactants [13,63]. The magnetite nanoparticles prepared with this method have dimensions in the 3 to 20 nm range adjusted by a control of the reaction time or the amount of the low complexing reactants. FeO(OH) has also been proposed as an organic precursor for thermal synthesis to produce nanoparticles with sizes below 20 nm [64]. A summary of the most relevant approaches using the thermal decomposition of organic precursors can be found in Table 1.

The article "Superparamagnetic Nanoparticles for Atherosclerosis Imaging" was published in 2014. Journal: Nanomaterials (Basel).

**Figure 2:** TEM images of 16-nm IONPs synthesized by the decomposition of organic precursors:  (**A**) a monolayer assembly; (**B**) a multilayer assembly; (**C**) High Resolution Transmission Electron Microscopy (HRTEM) image of a single Fe_3_O_4_ nanoparticle. Reproduced with permission from [13]. Copyright 2002, American Chemical Society.

**Table 1:** Main aspects of the synthesis of superparamagnetic iron oxide nanoparticles by thermal decomposition methods. PAA, polyacrylic acid.

Iron precursors	Surfactant	Solvent	T/°C	Shape and Size	Refs.
FeCup_3_	Octylamine	Trioctylamine	250–300 °C	4–10 nm	[15]
Fe(CO)_5_	Oleic acid	Dioctyl ether	300 °C	4–16 nm	[57]
Fe(CO)_5_	tri-n-octylphosphine oxide (TOPO)	Ortho-dichlorobenzene	180 °C	12 nm variation possible (diamond, triangle, spherical)	[67]
Fe(acac)_3_	Oleic acid Oleyl amine	Phenyl etheror benzyl ether	259–298 °C	<20 nm Seed mediated growth: 20 nm	[13] [63]
Fe(oleate)_3_ from FeCl_3_ and sodium oleate	Oleic acid	1hexadecane or trioctylamine or (2 more)	274–365 °C	5–22 nm	[61]
FeO(OH)	Oleic acid	1-octadecene	320 °C	6–30 nm	[64]
Fe(acac)_3_ FeCl_3_	2-pyrrolidone 2-pyrrolidone	2-pyrrolidone 2-pyrrolidone	245 °C	5 nm Seed mediated growth: 11 nm	[14] [13]
Fe(acac)_3_	m PEG-COOH d PEG-COOH	2-pyrrolidone 2-pyrrolidone	240 °C 240 °C	12–30 nm	[71] [72]
Fe(acac)_3_	PVP	*N*-vinyl-2-pyrrolidone	200 °C	4–40 nm	[73]
FeCl_3_	PAA	diethylenglycol	220 °C	3–12 nm	[74]

The size and morphology of the nanoparticles are the result of the growth mechanism during the thermal decomposition method. We will focus in this review only on the influence of the different reaction conditions; further details of the growth mechanism models have been reviewed in several occasions, like in Gao *et al* [65]. For instance, the time of reaction of the growth phase clearly regulates the size [66]. Furthermore, nanoparticles prepared with higher temperatures lead to larger sizes; successfully employed by heating with various solvents of high boiling points [61]. Another critical variable in the structural features of the nanoparticles is the surfactant or mixture used for emulsifying the systems and to control nucleation. It was observed that the size of the nanoparticles is inversely proportional to the tendency of the surfactant to coordinate with the iron atom [67,68]. Thus, common methods often control the size of the nanoparticles by the addition of a low complexing surfactant [68]. Sizes can also be modified depending on the molar proportion, Fe:surfactant [64]. Finally, it was shown that the affinity properties of the solvent for iron can play a major role in this process [69]. Although few studies also assessed the influence of the organic iron precursors, preliminary observations show that a narrower and controlled particle size distribution is favored with a specific iron intermediate complex before the generation of the cores [70].

The article "Superparamagnetic Nanoparticles for Atherosclerosis Imaging" was published in 2014. Journal: Nanomaterials (Basel).

Shape-controlled synthesis of iron oxide nanoparticles with this method can be performed under thermodynamic or kinetic control. Thermodynamic control is the key aspect when working with a low concentration of precursors, yielding spherical nanoparticles to minimize the surface energy. When working at high concentration conditions, kinetic control will lead to the formation of particles with other morphologies, such as cubic or elongated particles [62,69,75].

The above described thermal decomposition synthesis is a powerful method to produce IONPs of higher quality than the ones prepared by the aqueous routes [68]. One drawback of this approach is that the hydrophobic character of the nanoparticles makes compulsory a second step to transfer the IONPs to water. This necessity of rendering hydrophilic nanomaterials has boosted the appearance of new efficient chemical routes for the functionalization of nanoparticles.

Before the use of these new alternatives, the efforts focused on the modification of the thermal decomposition method with hydrophilic surfactants and/or polar solvents to provide hydrophilic nanoparticles in a one-pot synthesis route. Gao’s group first reported the use of 2-pyrrolidone, a strong polar organic solvent [14]. In the first attempt, 2-pyrrolidone had also the role of surfactant with Fe(acac)_3_ as the iron precursor. These nanoparticles of roughly 5 nm were hydrophilic, but with poor stability, being stable under acidic or alkaline conditions, which provides optimum electrostatic repulsion, but showed aggregation at neutral pH conditions. This method was assessed also with FeCl_3_∙6H_2_O as a precursor to obtain nanoparticles with an average size between 4 nm and 60 nm [76]. In order to synthesize nanoparticles stable in physiological solutions, mono- or di-carboxylic-terminated poly(ethylene glycol) (PEG) polymers were introduced as the surfactant [71,72]. The amphiphilic character of this PEG coating confers on iron oxide nanoparticles’ important properties, such as high stability and solubility in different media [14]. Moreover, di-substituted carboxylic polymers have the advantage of showing a reactive group on the surface for further functionalization. These results opened a range of new studies assessing others polar organic solvents and surfactants, such as polyacrylic acid (PAA), *N*-vinyl-2-pyrrolidone, glycols or diphenyl oxide [73,74,77,78].

The article "Superparamagnetic Nanoparticles for Atherosclerosis Imaging" was published in 2014. Journal: Nanomaterials (Basel).

### 2.3. Microwave-Assisted Synthesis

The use of microwaves in inorganic chemistry goes back to the 1970s and in organic chemistry to the 1980s. Although slow at the initial stages, the utilization of microwaves in chemical synthesis processes boosted from the mid-1990s. The main reasons for this increase included the availability of commercial equipment, the short reaction times and the expanded reaction range that is offered by microwave-assisted synthesis. These features make this approach particularly suited for the increased demands in industry.

In general, most of the synthetic reactions to obtain IONPs include heating through traditional heat transfer equipment, such as oil baths, sand baths and heating jackets. These heating techniques are, however, rather slow, and a temperature gradient can develop within the sample, leading to local overheating spots. All these parameters may have an important effect both in the nucleation and growing steps of the synthesis. A fundamental aspect of the microwave approach is the dielectric heating; under these conditions, the energy is introduced into the reactor remotely. The microwave radiation passes through the walls of the vessel and heats only the reactants and solvent and not the reaction vessel itself. In modern pressurized equipment, the temperature increase is uniform throughout the sample and facilitates heating far above the conventional boiling point of the solvent. All these features allow for the synthesis of IONPs with greater control/reproducibility of size and dispersity, as well as enhanced crystallinity.

The characteristics we just highlighted are attracting the attention of many scientists working in the synthesis of nanoparticles. Currently, there are examples in the literature of the use of microwaves for the synthesis of maghemite nanoparticles [33,34,35], mixed maghemite and magnetite nanoparticles [36] and pure magnetite [38]. Due to the novelty of the approach, most of the recent publications focused more on the synthesis of the nanoparticle core and rather poorly on the colloidal stability of the synthesized nanoparticles in water. This is gradually changing, and there are examples already using PEG and dextran as surfactants for biomedical applications [24,79,80]. Considering these data, it is not difficult to foresee in the near future a field where the utilization of microwaves for the synthesis of IONPs will be of paramount importance; for example, in the synthesis of dual PET/MRI nanoparticles, where not only the quality of the nanoparticles is important, but also the rapid incorporation of the radioisotope, particularly with those of reduced half-life isotopes (^18^F and ^68^Ga) [81]. The synthesis of this type of nanoparticles would be a clear improvement in comparison with traditional chelator-based compounds from the point of view of toxicity, no transmetallation *in vivo* and a much better biodistribution, provided the surface of the nanoparticles is properly functionalized [82].

The article "Superparamagnetic Nanoparticles for Atherosclerosis Imaging" was published in 2014. Journal: Nanomaterials (Basel).

## 3. Biofunctionalization of Iron Oxide Nanoparticles

When developing nanoparticles for biomedical or cardiovascular applications, the key point is the functionalization of the nanoparticles’ surface. Ideally, the functionalization should provide nanoparticles with very good colloidal stability in the usual conditions for *in vivo* administration (*i.e.*, 0.9% NaCl, PBS, *etc.*) and provide as many as possible functional groups that can be employed for the attachment of biomolecules.

The approach is different depending on the hydrophilic character of the initial IONPs. For those obtained by the coprecipitation method, the next step after the synthesis is the attachment of the biomolecule of interest. This sometimes can be a problem, since the number of functional groups on the surface is not that high. Since the IONPs obtained by thermal decomposition are usually of superior quality, we will focus this section on the functionalization of these particles.

Traditionally, for the stabilization of the hydrophobic nanoparticles synthesized by thermal decomposition, there were two main approaches: the micelle-like approach and the ligand exchange. Recently, a new approach has been developed by our group based on the direct chemical modification of the organic surfactant; something that presents a number of advantages [83,84,85,86].

### 3.1. Ligand Exchange

The ligand exchange approach is based on a mixture of hydrophobic IONPs with a very high concentration of the hydrophilic molecule. In such conditions, the hydrophilic ligand eventually displaces the hydrophobic surfactant, due to its affinity towards IONPs surface, thus yielding aqueous stable nanoparticles [87,88]. The most remarkable aspects of this approach are the simplicity and versatility, due to the enormous number of hydrophilic ligands that can be used for this purpose, like carboxylates, phosphates, polymers and inorganic materials (Table 2) [89,90,91,92,93,94]. However, this approach also presents some disadvantages. One of them is the degree of exchange. If this is not high, the surface of the nanoparticle will contain hydrophobic moieties, leading to stabilization problems and, most importantly, to a significant reduction in the number of reactive functional groups for further functionalization [95].

The article "Superparamagnetic Nanoparticles for Atherosclerosis Imaging" was published in 2014. Journal: Nanomaterials (Basel).

**Table 2:** Summary of the main properties for the most common ligand-exchange protocols. DMSA, dimercaptosuccinic acid; PAMAM, poly(amido)amine; PAH, poly(allylamine).

Ligand	TEM (nm)	DLS ^1^ (nm)	*r*_2_ (mM^−1^s^−1^)	Ref.
DMSA	9.0 ± 2.0	65.0 ± 5.0	317	[103]
Citric acid	4.0 ± 0.5	8.6 ± 1.0	33	[56]
1-mercapto-11-undecanoic acid	10.0 ± 3.0	170.0 ± 50.0	n.a.	[104]
2-bromo-2-methylpropionic acid	8.0 ± 1.0	n.a.	n.a.	[105]
PEG-SiMe3	8.4 ± 1.5	12.2 ± 2.7	n.a.	[98]
NH2-SiMe3	8.7 ± 1.3	14.4 ± 2.8	n.a.	[98]
COOH-SiMe3	8.2 ± 1.2	13.5 ± 2.0	n.a.	[98]
Hydroxyethylenebisphosphonate	5.0 ± 1.5	15.2 ± 2.5	122	[101]
Stilbenephosphonate	6.0 ± 0.5	39.0 ± 5.0	n.a.	[106]
PMIDA ^2^	5.0 ± 0.5	62.0 ± 3.0	n.a.	[107]
PAMAM	5.0 ± 2.0	90.0 ± 20.0	79	[108]
Melanin-Dopamine	10.0 ± 2.0	n.a.	114	[109]
PAA-PAH	11.0 ± 2.0	60.0 ±10.0	n.a.	[110]
PNIPAM-b-PNIPAM ^3^	15.0 ± 3.0	60.0 ± 4.0	n.a.	[111]
DPA ^4^-PEG-COOH	9.0 ± 1.0	40.0 ± 2.0	n.a.	[112]

^1^ DLS: Dynamic Light Scattering; ^2^ PMIDA: *N*-phosphonomethyl iminodiacetic acid; ^3^ PNIPAM: Poly(*N*-isopropylacrylamide); ^4^ DPA: methacrylate-co-2-(diisopropylamino)ethyl methacrylate.

In general, the ligands utilized in this approach can be classified as small organic molecules and large polymeric compounds, such as dimercaptosuccinic acid (DMSA). This ligand, due to the carboxylic groups, shows a high affinity towards the IONP surface, thus providing high stability in aqueous media and enough free functional groups for further biomolecule conjugation with many applications [77,96,97]. DMSA-nanoparticles, with a small hydrodynamic size (less than 50 nm) and very good magnetic properties, can be obtained with this approach. These nanoparticles can be employed, for instance, for MRI and also drug delivery. Citric acid is another carboxylic-based ligand for the ligand exchange approach of common use in this very field. This acid may be adsorbed on the surface of the magnetite nanoparticles via one of the two carboxylate groups, depending on steric hindrance and the curvature of the surface. This leaves at least one of these functional groups exposed to the solvent, which should be responsible for making the surface negatively charged and hydrophilic [56].

The article "Superparamagnetic Nanoparticles for Atherosclerosis Imaging" was published in 2014. Journal: Nanomaterials (Basel).

Another kind of ligand with good properties for the exchange approach are silanes (Figure 3). These compounds present the general chemical formula, X-(CH_2_)_n_-SiR_3_, where SiR_3_ is the anchor group having good affinity for the surface of the nanoparticle, (CH_2_)_n_ is the hydrophobic chain and X is the headgroup providing the hydrophilicity. Further surface modifications are possible depending on the X group [98]. The efficiency of ligand exchange reactions with silanes depends on various factors, like the concentration of the silicon tetrahydride, the reaction times and the presence of a catalyst [99]. Although ligand exchange is a straightforward method and these factors can be easily controlled, the method with silanes shows poor reproducibility [100]. Other small molecules that have been used in this approach are phosphonates, of several compositions [101,102].

The utilization of large polymeric compounds for the exchange approach includes dendrimers, polyacrylic acid and PEG. In the case of dendrimers, the most common of these molecules in biomedicine, poly(amido)amine (PAMAM), is also the most commonly used for the functionalization of IONPs. These dendrimers have been conjugated with targeting ligands, imaging moieties and drug molecules for its application in cancer therapy [108,113,114]. Moreover, poly(amido)amine IONPs are a suitable platform for further functionalization to increase the circulation time of the nanoparticles in blood [51]. These macromolecules are obtained via conventional organic synthesis. In this regard, maghemite nanoparticles with uniform and monodisperse sizes were functionalized with dopamine, showing good aqueous stabilization [109].

**Figure 3:** Structure of common silane-based molecules for the ligand exchange approach.

Polyelectrolytes, such as poly(acrylic acid) (PAA) and poly(allylamine) (PAH), are employed to replace the original hydrophobic ligands on the surface of iron oxide nanoparticles. These polymers need high temperature in ligand exchange reactions with IONPs. Therefore, polar solvents with a high boiling point, like diethylene glycol, are commonly used. Moreover, diethylene glycol has high miscibility in both aqueous and typical organic solvents and high power to dissolve polyelectrolytes, providing good features for this type of ligand exchange reaction with polymers at high temperature (>240 °C). In the case of PAA-PAH, nanoparticles, with a narrow core size distribution, stability in water and good magnetic properties, are obtained in a short reaction time [110].

The article "Superparamagnetic Nanoparticles for Atherosclerosis Imaging" was published in 2014. Journal: Nanomaterials (Basel).

As we have mentioned before, nanoparticle PEGylation with chains of different molecular weight, is well established to optimize the stabilization of nanoparticles and to prolong their circulation time in blood after administration [115,116,117]. Regarding the utilization of this polymer in the ligand exchange approach, one of the best examples is the use of DPA-PEG-COOH (DPA: methacrylate-co-2-(diisopropylamino)ethyl methacrylate), a synthetic compound produced from polyethylene glycol diacid (HOOC-PEG-COOH), in which one of the acid groups reacts with the terminal free amine of dopamine through the conventional EDC/NHS (1-Ethyl-3-(3-dimethylaminopropyl)carbodiimide/*N*-Hydroxysuccinimide) reaction obtaining DPA-PEG-COOH. After a ligand exchange reaction among DPA-PEG-COOH and oleic acid nanoparticles, water stable nanoparticles are achieved, even with different length chains of PEG. These nanoparticles have proven to have much less uptake by macrophages, indicating that these can evade recognition from these cells of the immune system [112].

### 3.2. Micelle-Like Approach

**Figure 4:** Micelle approach for PAMAM-C12 coating of the oleic acid-capped iron oxide nanoparticles. Reproduced with permission from [142]. Copyright 2013, American Chemical Society.

The utilization of amphiphilic structures for the stabilization and functionalization of IONPs is a second approach usually selected when synthesizing these compounds [118,119,120,121,122]. This method takes advantage of the structure of these amphiphilic molecules. The formation of weak van der Waals interactions between the hydrophobic part of these molecules and the organic tail of the nanoparticle coating, to minimize the interaction with water, produces very stable nanoparticles with excellent reproducibility (Figure 4). Furthermore, the possibility of a previous modification on the amphiphilic molecule allows for the stabilization and functionalization of the IONPs to be carried out in a single step, although this opportunity has not been fully addressed. To obtain such micelle-like structures, usually, the first option is to use a polymeric amphiphilic compound. The hydrophobic structure is inserted between the hydrophobic chains of the surfactant/ligand adsorbed on the nanoparticle, while the hydrophilic part stands around the outer surface to assure the dispersion of the IONPs in biological media. Many kinds of polymers have been assessed, like pluronic [123,124,125,126], poly(maleic anhydride alt-1-tetradecene) [127], cyclodextrins [128], PEG-phospholipids conjugates [129,130] or other triblock polymers [131,132,133]. Other advantages of the method are the possibility of further crosslinking for better stabilization or encapsulation of small hydrophobic drugs in the hydrophobic bilayer that is created (as well as small organic fluorescent molecules). The final stability of the structure depends mainly on the nature of the polymers, *i.e.*, amphiphilic balance, molecular weight, length of the chains or conformation [131].

The article "Superparamagnetic Nanoparticles for Atherosclerosis Imaging" was published in 2014. Journal: Nanomaterials (Basel).

To achieve the insertion of the polymers, several methods are possible, such as reverse evaporation [134,135], progressive increase of the solvent polarity [131] or nanoemulsion [136]. The encapsulation of hydrophobic nanoparticles in polymeric micelles [137] is very similar to the insertion option. Many examples are in the bibliography using diblock polymers, such as polylactide-b-poly(ethylene-maleimide) [122,138], poly(styrene-block-acrylic acid) [131], poly(e-caprolactone)-b-poly(ethylene glycol) [139,140] or dendrimers [141].

Control of self-assembly structures can be achieved from micelles to vesicles, based on the nature of the solvent used and other conditions [133]. Liposomes are another important structures based on amphiphilic compounds. Liposomes are vesicles composed of a lipid bilayer, and a very important platform for drug delivery and imaging applications [143]. To explain in detail the utilization of liposomes in general or their application in the synthesis of iron oxide nanoparticles, one will need another review, so we refer the reader to other sources already dealing with this aspect in detail, particularly those by Torchilin *et al.* in 2005 and Alen *et al.* in 2013 [142,143,144,145,146,147]. Here, we will only mention one work, especially relevant for the topic covered in this review, by Fayad and Mulder *et al.* (Figure 5) [148]. In this work, an HDL-like nanoparticle (HDL, high density lipoprotein) was developed with multimodal imaging properties, by including additional labels in the corona of the particles, such as iron oxide, Au and quantum dots. The *in vitro* and *in vivo* characterization of these particles demonstrated that they mimic many of the properties of the native HDL and, therefore, could be used for *in vivo* imaging of atherosclerotic plaque.

**Figure 5:** Schematic structure and TEM imaging of HDL-iron oxide nanoparticles. Adapted with permission from [149]. Copyright 2008, American Chemical Society.

### 3.3. Chemical Modification of the Surfactant

One of the new approaches that we review is based on the direct chemical modification of the surfactant, usually oleic acid. The ligand exchange method is based on the partial replacement of the oleic acid, whilst the micelle approach focuses on keeping it, but hidden below at least under a layer of the amphiphilic molecules. The chemical modification approach is based instead on performing organic reactions over the oleic acid. The final intention of this method is to bring all organic chemistry tools for the synthesis and functionalization of hydrophilic molecules. Although different alternatives can be foreseen, the most logical one is to perform chemistry in the functional group of oleic acid that is not involved in the surface binding of the nanoparticles: the carbon-carbon double bond. So far, there are two strategies that have been followed in this approach (Figure 6). 

The article "Superparamagnetic Nanoparticles for Atherosclerosis Imaging" was published in 2014. Journal: Nanomaterials (Basel).

**Figure 6:** Direct chemical modification of the surfactant for oleic acid-coated IONPs, by (**A**) oxidation of the double bond and (**B**) olefin metathesis by the use of Hoveyda-Grubbs 2nd generation catalyst.

We have demonstrated this approach for the first time in iron oxide nanoparticles, by using the very well-known double-bond oxidation with KMnO_4_ to generate a carboxylic group (Figure 6A). It is known that under these conditions, the permanganate ion forms a complex with the double bond that can be hydrolyzed in both acidic and basic pH. Under these conditions, IONPs were obtained with a 40 nm mean diameter, a zeta potential of −46 mV and good magnetic (Ms = 77 emu/g Fe) and relaxometric properties (*r*_1_ and *r*_2_ are 4 s^−1^ mm^−1^ and 115 s^−1^ mm^−1^). The reaction is performed in a two-phase system, a mixture of organic solvent, where the oleic acid nanoparticles are dispersed, and an aqueous phase, where the KMnO_4_ is soluble and where the IONPs are eventually dispersed. In this procedure, a phase-transfer catalyst is used to get enough concentration of the MnO_4_^−^ ion in the organic phase. The best results are obtained usually with trimethylbenzylammonium chloride.

This modification renders water-stable particles and, at the same time, also, a functional group ready for the further attachment of biomolecules, from small organic molecules to dyes and proteins [84,85] (Figure 7). Two of the most remarkable features of these modifications are that the nanoparticle is always protected by a layer of surfactant, thus minimizing the aggregation and that, by using an excess of the oxidant, a complete transformation of the oleic acid is achieved, as we demonstrated using magnetic resonance spectroscopy, mass spectrometry and infrared. This is a very important difference compared to the previous methods. By removing all oleic acid from the surface, more stable nanoparticles and less toxicity problems are expected. The same is true for further functionalization, since this approach allows for strong covalent interaction that, at no point, exposes the core of the nanoparticle [83,150].

The article "Superparamagnetic Nanoparticles for Atherosclerosis Imaging" was published in 2014. Journal: Nanomaterials (Basel).

**Figure 7:** Synthesis of multifunctional IONPs by the direct chemical modification of oleic acid. The attachment of allergen Phl p5a and a fluorophore, via biotin-streptavidin interaction, was done by amide formation with the carboxylic groups generated. TEM image of the final IONPs (**bottom** **left**). Immunogenicity of the synthesized nanoparticles compared to non-functionalized particles, grass pollen extract and pure protein (**bottom** **right**). Reproduced from [87]. Copyright 2012, John Wiley & Sons, Ltd.

A second recent initiative is the direct modification of oleic acid using another well-known reaction in organic chemistry, the olefin cross-metathesis. The idea behind this is to take advantage of the functional group in the oleic acid. However, with the olefin metathesis option, we can go one step further. Since it is possible to incorporate a terminal olefin in many proteins and biomolecules, it can be utilized for, in a single step, transferring the nanoparticles to water and providing specificity for biomedical applications [86,149,151]. Using this method, biofunctionalized IONPs are obtained again in two steps, but with better physicochemical properties.

## 4. Application to Atherosclerotic Plaque

Atherosclerosis is an inflammatory pathology of the blood vessel wall in which plaque builds up inside the arteries [152,153,154,155,156]. Plaque is mainly made up of lipids, cholesterol, calcium, macrophages and several substances found in the blood. Over time, plaque hardens and narrows the arteries, limiting the flow of oxygen-rich blood to the organs.

During the atherothrombotic plaque formation, relevant events take place: inflammation, deposition of cholesterol, extracellular matrix (ECM) development and thrombosis [157,158,159]. Characteristics of atherosclerosis are the presence of fibrous and lipid-rich elements in vessel walls of arteries (coronary, carotid and aorta as the most common injured arteries). During the course of the pathology, myeloid cells de-stabilize the plaque, causing it to rupture [160]. Most of the damage occurs when plaques become fragile and rupture. Plaques that rupture cause the formation of blood clots that can block blood flow or break off and travel to another part of the body. Monocytes are infiltrated during early damage in the arterial wall and, in combination with macrophages, promote the inflammatory process. After activation of macrophages from monocytes in the sub-endothelial space, the ingestion of high amounts of lipids by the activated macrophages triggers the origin of foam cells. The accumulation of lipid cores by foam cells activated macrophages and necrotic cells, leading to the migration of smooth muscle cells to intima, forming the fibrous cap over the damage (Figure 8). These inflammatory events’ expression, accompanied with the delivery of proteolytic enzymes (metalloproteinases, cysteinyl cathepsins), which catabolize the extracellular matrix of fibrous cap in plaques, are responsible for plaque instability [161]. When this fibrous cap becomes thin, the plaque vulnerability risk is increased [152]. The complete mechanism explaining plaque instability and proneness to rupture is unknown yet [156].

The article "Superparamagnetic Nanoparticles for Atherosclerosis Imaging" was published in 2014. Journal: Nanomaterials (Basel).

### 4.1. Molecular Imaging in Atherosclerosis

One of the main issues of an atherosclerotic lesion is that it develops slowly over decades, being finally identified at advanced states of the pathology [155]. One of the main goals in the utilization of molecular imaging in atherosclerosis is the possibility of early diagnosis, at a subclinical point [162,163].

Current approaches in atherosclerotic plaque imaging are mainly based on molecular imaging approaches by the targeting of biomolecules involved in the lesion progression. Macrophages are one of the most utilized targets in molecular imaging, due to their role during inflammation [152,156,163]. However, there are important biochemical targets that are indicative of plaque development, such as metalloproteinases, LDL-oxidized, calcium vesicles or receptors involved in neoangiogenesis [152,155,156]. Molecules involved in plaque rupture, like metalloproteinases (MMPs) and cathepsins, are highly recommended as molecular imaging targets.

**Figure 8:** Evolution of atherosclerosis disease and the main targets at each step, according to the American Heart Assocciation (AHA). Reproduced with permission from [158]. Copyright 2008, Nature Publishing Group.

### 4.2. Iron Oxide Nanoparticles in Atherosclerosis Imaging

The use of IONPs for atherosclerosis targeting makes use of the principal markers of the disease, such as MMPs, angiogenesis, activated platelets, cell adhesion molecules, apoptosis markers and fibrin markers. The first results with IONPs as a platform for molecular imaging in this context comes from the rapid uptake by the macrophages of the immune system [164,165,166,167,168]. Systematic evaluation of MRI with IONP as a contrast agent in carotid atheroma confirmed that the optimal signal intensity was achieved 24–36 h after i.v. (Intravenous) administration. In 2000, it was demonstrated that there is a spontaneous phagocytic uptake of superparamagnetic iron oxide nanoparticles by macrophage populations in atherosclerotic plaque [164,169]. There are numerous examples showing the feasibility of atherosclerosis imaging by the non-specific labeling of macrophages [162,163,170]. This has been done, for example, in humans, with IONPs synthesized by the coprecipitation approach and coated with dextran [168]. This study showed that the nanoparticles accumulate predominantly in macrophages in ruptured and rupture-prone human atherosclerotic lesions, inducing significant signal changes in the *in vivo* T2*w fast gradient echo MRI. Similar results were obtained later, also in humans, with the same type of nanoparticles in the imaging of carotid atheroma. The nanoparticles accumulated in macrophages of seven out of eight patients, demonstrating areas of MRI signal reduction that correspond to IONPs/macrophage-positive histological sections. The MRI signal change was obtained between 24 h and 36 h after injection and was still evident up to 96 h after infusion. The explanation of how the IONPs are phagocytized by macrophages and end up in the plaque is related to the endothelial dysfunction theory. Plasma components are accumulated in the sub-endothelial space, allowing the progression of arterial wall inflammation. Low-density lipoproteins (LDL) are accumulated in their oxidized form and then phagocytized by macrophages. Finally, they form foam cells. The main similarity between LDL and IONPs are the diameter size (15–25 nm) and capability of accumulation in atheroma plaque with high macrophage activity [170]. Pharmacokinetics and the specific biodistribution of the probes based on IONPs depends on the particle size, as well as on the charge and surface properties [152,156,170,171]. Smaller particles are less efficiently uptaken than larger particles in the case of phagocytic cells.

The article "Superparamagnetic Nanoparticles for Atherosclerosis Imaging" was published in 2014. Journal: Nanomaterials (Basel).

Another important option for the use of IONPs in atherosclerosis is the binding of specific ligands on the surface of the particles to increase selectivity. This has been done also for the labeling of macrophages; for example, with the binding of the PP1 LSLERFLRCWSDAPAK peptide that binds to SR-A receptors. These belong to the scavenger receptor family, which has an important role during foam cell formation and consequent activation. Increased expression of these receptors has been reported in foam cells during atherosclerotic damage and vascular smooth muscle cells (VSMCs) after plaque inflammation events [163,172]. It is possible to conjugate this ligand to the IONPs in order to increase nanoparticle uptake. A significant increment of this PP1-conjugated IONPs *in vitro* using plaque-associated macrophages and VSMCs was reported [172]. Similar results of nanoparticle accumulations were obtained by contrast-based MRI in atherosclerotic plaque lesions with humanized models using Western-type diet-fed LDLR^−/−^ with human SR-AI, and in aged models with ApoE^−/−^ mice [163].

The article "Superparamagnetic Nanoparticles for Atherosclerosis Imaging" was published in 2014. Journal: Nanomaterials (Basel).

Other important targets are cell adhesion molecules. Among them, due to its strict temporal and spatial expression/regulation, VCAM-1 has received most of the attention. There are several studies involving ligand-conjugated IONPs for MRI of endothelial adhesion molecules (VCAM-1 and P-selectin) [173,174]. IONPs have been conjugated with VCAM-1 internalizing peptides, identified by phage display. It has been reported that they are accumulated by cells with upregulated expression of VCAM-1, being specific for activated endothelium [153,156,173,174]. With the same aim of monitoring these proteins, IONPs could be also conjugated to specific moieties, like MHC-I peptides and VCAM-1 antibodies [156]. Another possible candidate is P-selectin, which is overexpressed on pathologically activated endothelium surfaces and activated platelets during atherosclerosis initiation, progression, rupture and thrombosis [175]. This marker has in fact been used for the synthesis of IONPs conjugated to an antihuman P-selectin antibody (VH10). The nanoparticles were validated in a model with ApoE^−/−^ mice using a bimodal magnetofluorescent agent, for MRI and optical imaging of an inducible P-selectin expression in human activated platelets involved in the early stages of atherosclerosis [176]. Apoptosis is another event during plaque destabilization that has been used for the selective accumulation of IONPs in the atheroma lesion by the attachment of Annexin V in the surface of these nanoparticles. It is known that this protein has a high binding affinity for phosphatidylserine residues, translocated to the outer leaflet of the plasma membrane in apoptotic cells. The selective accumulation of such nanoparticles in atherosclerosis models in rabbits was shown by MRI [177].

Fibrin is also a good target for atherosclerosis detection with IONPs. Using a thermal decomposition approach, Sepan *et al.* prepared iron oxide nanoparticles coated with specific functional groups of fibrin by the nanoemulsion method (Figure 9), obtaining a micelle-like nanostructure. These nanoparticles were tested using T1 weighted imaging, which is far much easier to identify *in vivo* [178].

**Figure 9:** Fibrin-specific IONPs for the T1-weighted imaging of fibrin in atherosclerotic plaque. Reproduced with permission from [178]. Copyright 2009, American Chemical Society.

As a final example, we would like to highlight a recent contribution that makes use of one of the very well-known nanoparticles [179], IONPs coated with citric acid, which show selective accumulation in the calcifying microvesicles, characteristics of the atheroma lesion and also, to some extent, in the activated macrophages. All this makes these nanoparticles good candidates as probes for the study of the composition and inflammatory activity of the plaque at risk of destabilization.

The article "Superparamagnetic Nanoparticles for Atherosclerosis Imaging" was published in 2014. Journal: Nanomaterials (Basel).

## 5. Conclusions

The utility of nanotechnology in the study of cardiovascular diseases is currently fully demonstrated, from diagnosis to therapy. From the examples we have shown, it is clear that there are many examples of iron oxide-based particles able to diagnose and/or treat the atheroma plaque. For the next few years, the most difficult aspect that must be addressed is the applications of these nanoparticles in the clinic. For that to happen, one of the most important aspects is the development of reliable and reproducible methodologies allowing for the synthesis of the targeted nanoparticles we just saw. In our opinion, the best chances of achieving this goal is with the development of bio-orthogonal or chemo-selective approaches for the coupling of biologically-relevant compounds or drugs on the surface of IONPs. This kind of chemistry can deliver nano-compounds with controlled and specific composition on the surface. Moreover, it will allow for the binding of biomolecules with their intact native structure and function, assuring the best performance in terms of molecular imaging and disease treatment. This last point will also mean a clear advantage over the use of radionuclide-based probes for atherosclerosis, since, with a single radiation-free probe, the diagnosis, therapy and follow-up of the disease could be achieved. We consider that in the coming years, we will assist in the boom of this kind of functionalized nanoparticles in the field of cardiovascular imaging.
